RETRACTED

# Analysis of Risk Factors for Intraoperative Hypotension in Cesarean Section and Poor Prognosis of Neonates

**DOI:** 10.1155/2022/2468114

**Published:** 2022-03-24

**Authors:** Yang Liu, Yanning Qian

**Affiliations:** ^1^Department of Anesthesiology, The Affiliated Jiangning Hospital of Nanjing Medical University, No. 169, Hushan Road, Dongshan Street, Jiangning District, Nanjing 211103, China; ^2^Department of Anesthesiology, The First Affiliated Hospital with Nanjing Medical University, No. 300 Guangzhou Road, Nanjing 210029, China

## Abstract

**Objective:**

To analyze the risk factors of intraoperative hypotension in cesarean section women and poor prognosis of neonates.

**Methods:**

The clinical data of 1071 cesarean section women admitted to The Affiliated Jiangning Hospital of Nanjing Medical University from January 2021 to December 2021 were retrospectively analyzed. They were divided into hypotension group (*n* = 472) and normal control group (*n* = 599) according to whether there was hypotension during operation. The correlations between the clinical data of cesarean section and the occurrence of intraoperative hypotension and poor prognosis of neonates were analyzed by logistic regression analysis. Receiver operating curve (ROC) was drawn and the area under the curve (AUC) was calculated.

**Results:**

Logistic regression analysis results showed that BMI ≥30 kg/m^2^, infant weight ≥3500 g, spinal anesthesia, puncture site L_2-3_, bupivacaine dose>10 mg, ropivacaine dose>50 mg, and perfusion index≥4 were the risk factor for intraoperative hypotension in cesarean section (*p* < 0.01) and BMI ≥30 kg/m^2^, umbilical cord around neck, spinal anesthesia, and perfusion index≥4 were risk factors for poor prognosis of neonates (*p* < 0.01). The AUC of ROC for BMI to diagnose intraoperative hypotension in cesarean section women was 0.6240 (95% CI: 0.59-0.66, *p* < 0.01), the sensitivity was only 30.20% (95% CI: 26.73%-35.02%), and the specificity was 87.65% (84.77%-90.04%), and the AUC of BMI for the diagnosis of poor prognosis of neonates was 0.5647 (95% CI: 0.5013-0.6280, *p* = 0.049), and the sensitivity was 51.19% (95% CI: 40.69%-61.59%), and the specificity was 64.34% (61.30%-67.26%). The AUC of perfusion index for the diagnosis of intraoperative hypotension in cesarean section women was 0.8333 (95% CI: 0.8081-0.8584, *p* < 0.01), the sensitivity was 94.49% (95% CI: 92.05%-96.21%), and the specificity was 73.12% (69.43%-76.52%); the AUC of perfusion index for the diagnosis of ROC with poor prognosis of neonates was 0.6164 (95% CI: 0.5538-0.6791, *p* < 0.01), the sensitivity was 70.24% (95% CI: 59.75%-78.96%), and the specificity was 50.86% (47.75%-53.97%).

RETRACTED

**Conclusion:**

The prediction model established by BMI, infant weight, anesthesia method, puncture site, anesthetic drug dose, and perfusion index has guiding value for clinical prediction of cesarean section maternal hypotension. The prediction model established by BMI, umbilical cord around neck, anesthesia method, and perfusion index has guiding value for clinical prediction of poor prognosis of neonates.

## 1. Introduction

Cesarean section is a common surgical procedure around the world, and spinal anesthesia is one of the most commonly used anesthesia in cesarean section [1–3]. Compared with epidural anesthesia, spinal anesthesia can provide a better and lower cost anesthesia method for elective cesarean section [4]; however, the risk of complications such as hypotension after spinal anesthesia is higher, and persistent hypotension can lead to hypoperfusion of the placenta, which is prone to fetal distress, acidosis, and low Apgar score [5–7]. Therefore, how to reduce the risk of hypotension after spinal anesthesia during cesarean section surgery is one of the key topics in clinical research.

At present, there are many studies on hypotension after cesarean section anesthesia. In a study of risk factors for neonates with an Apgar score <7, the researchers found that emergency cesarean delivery, doses of the anesthetic ephedrine >30 mg, and a drop of more than 10% in diastolic blood pressure were risk factors for hypotension after cesarean section anesthesia. A systematic study reported a significant reduction in the risk of hypotension when the spinal anesthetic bupivacaine was administered at doses of 8 mg or less (hazard ratio: 0.78, 95% confidence interval: 0.65-0.93), [8]. In a study of 200 cesarean section women who underwent spinal anesthesia, hypotension occurred in about 70% of the patients; they believed that baseline systolic blood pressure >130 mmHg and pupillary response latency >223 ms were associated with risk of spinal anesthesia-related hypotension [9].

In this study, we analyzed the risk factors of intraoperative hypotension in cesarean section women and poor neonatal prognosis, and provided a basis for preventing the occurrence of intraoperative hypotension in cesarean section women and reducing the incidence of poor prognosis of neonates.

## 2. Materials and Methods

### 2.1. Subjects

The medical data of 1407 puerperae who underwent cesarean section in The Affiliated Jiangning Hospital of Nanjing Medical University from January 2021 to December 2021 were collected. A total of 336 patients were excluded, including 108 patients with cardiovascular disease, 302 patients with endocrine system diseases, and 22 patients with placenta previa, and finally a total of 1071 patients were included. The collected clinical information included age, American Society of Anesthesiologists (ASA) classification, body mass index (BMI), gestational age, gravidity, parity, gender, fetal position, uterine height, abdominal circumference, biparietal diameter, femoral length, fetal abdominal circumference, amniotic fluid index, the ratio of fetal umbilical artery systolic blood pressure to diastolic blood pressure (S/D), anemia, hypoalbuminemia, infant weight, umbilical cord around neck, incision direction, anesthesia type, puncture site, local anesthetic dose, occurrence of intraoperative hypotension, preoperative HR, preoperative mean arterial pressure (MAP), intraoperative blood loss, time from skin incision to delivery, perfusion index, pH value of umbilical artery blood, and 1-minute Apgar score. The flow chart of this study is shown in Figure 1.

RETRACTED

### 2.2. Inclusion and Exclusion Criteria

Inclusion criteria: (1) Cesarean section women with intraspinal anesthesia and the sensory block level reaches T_5-6_. (2) American Society of Anesthesiologists (ASA) Class I or II. (3) The fetus produced is a live fetus. (4) Gestational age ≥30 weeks. (5) Singleton pregnancy. Exclusion criteria: (1) Patients with cardiovascular disease. (2) Patients with endocrine system diseases. (3) Placenta previa. (4) Emergency cesarean delivery cases.

### 2.3. Anesthesia Method

Before surgery, the anesthesiologist should have a comprehensive understanding of the maternal condition, in order to make a correct assessment of the mother and the fetus, use an appropriate anesthesia method, ensure the safety of the mother and the fetus, and reduce surgical trauma and postoperative complications. Elective cesarean section women should fast for 6-8 hours and avoid drinking fluids for 4 hours before anesthesia. Before anesthesia, 500 ml of lactic acid forest solution was added, and a puncture needle with a finer type (25G and below) was selected. The patients were uniformly punctured in the L_2-3_ space or L_3-4_ space in the chest-knee position. After the outflow of cerebrospinal fluid, 0.5% bupivacaine (2 ml 0.75% bupivacaine + 1 ml normal saline mixture 3 ml) was injected into the subarachnoid space, and the injection rate was 0.1 ml/s. With epidural anesthesia, the anesthesiologist injected 0.5% ropivacaine intrathecally at a dose of 40-80 mg using an injection rate of 0.1 ml/s depending on the patient's condition. After anesthesia, the puerpera was placed in a supine position and the operating table was adjusted to a left tilt of 30°.

### 2.4. Criteria for Hypotension and Poor Prognosis of Neonates

The criteria for hypotension: MAP decrease >20% or SBP <90 mmHg [10–12]. Criteria for poor prognosis of neonates: Apgar score 1 min ≤7 and umbilical artery blood pH <7.2 [13, 14]. When hypotension occurred during surgery, 2 mg dopamine was given intravenously, but when the patient's heart rate was below 55 beats/min, 0.5 mg atropine was given intravenously.

RETRACTED

### 2.5. Statistical Analysis

In this study, IBM SPSS Statistics (version 26.0) was used for statistical analysis. Continuous variables that conformed to a normal distribution were expressed as mean ± standard deviation, and continuous variables that did not conform to the normal distribution were expressed as median [Q25, Q75]. The variables with statistical significance in the univariate variable analysis were included in the multivariate analysis, and the multivariate analysis used binary logistic regression to analyze the risk factors of intraoperative hypotension and poor prognosis of neonates in cesarean section women. The receiver operating curve (ROC) was used to analyze the diagnostic value of anesthetic drug dose and perfusion index in intraoperative hypotension and poor prognosis of neonates in cesarean section women. All tests were two-tailed and *p* <0.05 indicated a statistically significant difference.

## 3. Results

### 3.1. Clinical Information

The basic information of the cesarean section women in this study is shown in Table 1. The maternal age distribution was 18-47 years old, the body mass index (BMI) was 16.28-39.35 kg/m^2^, the gestational week was 31-41 weeks, 44.07% of the puerperae had hypotension during the operation, and up to 66.57% of the fetuses were located on the left side. The fetal weight was 1580-5190 g, and 7.84% of newborns had a 1-minute Apgar score below 7 after birth.

S/D: the ratio of fetal umbilical artery systolic blood pressure to diastolic blood pressure; MAP: mean arterial pressure; HR: heart rate.

### 3.2. Univariate Logistic Regression Analysis of Risk Factors for Hypotension during Cesarean Section

Logistic regression was used to analyze the risk factors of intraoperative hypotension in cesarean section women. The results are shown in Table 2. The results showed that BMI, infant weight, anesthesia type, puncture site, bupivacaine dose, ropivacaine dose, and perfusion index were associated with the occurrence of intraoperative hypotension in cesarean section women (*p* < 0.05).

S/D: the ratio of fetal umbilical artery systolic blood pressure to diastolic blood pressure; MAP: mean arterial pressure; HR: heart rate.

### 3.3. Multivariate Logistic Regression Analysis of Risk Factors for Hypotension during Cesarean Section

Regression analysis was performed with statistically significant factors as independent variables and whether hypotension occurred during cesarean section as dependent variable. The results showed that BMI ≥30 kg/m^2^, infant weight ≥3500 g, spinal anesthesia, puncture site L_2-3_, bupivacaine dose>10 mg, ropivacaine dose>50 mg, and perfusion index ≥4 were risk factors for intraoperative hypotension in cesarean section women (*p* < 0.01) (Table 3).

RETRACTED

### 3.4. Analysis of Risk Factors for Poor Prognosis of Neonates

Univariate logistic regression was used to analyze risk factors for poor prognosis of neonates (Table 4). The results showed that BMI, gestational age, parity, umbilical cord around the neck, anesthesia type, puncture site, intraoperative hypotension, time from skin incision to delivery, and perfusion index were associated with poor prognosis of neonates (*p* < 0.05).

Regression analysis was performed using factors with statistically significant differences in univariate analysis results as independent variables and poor neonatal prognosis as dependent variable. The results showed that BMI ≥30 kg/m^2^, umbilical cord around neck, spinal anesthesia, and perfusion index ≥4 were risk factors for poor prognosis of neonates (*p* < 0.01) (Table 5).

### 3.5. ROC of BMI and Perfusion Index for the Diagnosis of Intraoperative Hypotension and Poor Neonatal Prognosis in Cesarean Section Women

The ROC was used to analyze the diagnostic value of BMI and perfusion index in the diagnosis of intraoperative hypotension and poor neonatal prognosis in cesarean section women. The results showed that the AUC of the ROC for BMI to diagnose intraoperative hypotension in cesarean section was 0.6240 (95% CI: 0.5900-0.6600, *p* < 0.01), and the cut-off value was 32.80 kg/m^2^, but the sensitivity was only 30.20% (95% CI: 26.73%-35.02%), and the specificity was 87.65% (84.77%-90.04%) (Figure 2(a)). The AUC of BMI to diagnose poor neonatal prognosis was 0.5647 (95% CI: 0.5013-0.6280, *p* = 0.049), the cut-off value was 29.75 kg/m^2^, and the sensitivity was 51.19% (95% CI: 40.69%-61.59%), and the specificity was 64.34% (61.30%-67.26%) (Figure 2(b)).

The AUC of perfusion index for the diagnosis of intraoperative hypotension in cesarean section women was 0.8333 (95% CI: 0.8081-0.8584, *p* < 0.01), the cut-off value was 5.845, and the sensitivity was 94.49% (95% CI: 92.05%-96.21%), the specificity was 73.12% (69.43%-76.52%) (Figure 2(c)). The AUC of perfusion index for the diagnosis of poor neonatal prognosis was 0.6164 (95% CI: 0.5538-0.6791, *p* <0.01), the cut-off value was 6.405, and the sensitivity was 70.24% (95% CI: 59.75%-78.96%), and the specificity was 50.86% (47.75%-53.97%) (Figure 2(d)).

RETRACTED

Therefore, BMI cannot be used to predict the occurrence of intraoperative hypotension and poor neonatal prognosis in cesarean section women. The perfusion index is a potentially valuable indicator of intraoperative hypotension in cesarean section, but the perfusion index is not specific for poor neonatal prognosis.

## 4. Discussion

In this study, we analyzed the risk factors for intraoperative hypotension and poor neonatal prognosis in cesarean section women; the results showed that BMI ≥30 kg/m^2^, infant weight ≥3500 g, spinal anesthesia, puncture site L_2-3_, bupivacaine dose>10 mg, ropivacaine dose>50 mg, and perfusion index ≥4 were risk factors for intraoperative hypotension in cesarean section women, and BMI ≥30 kg/m^2^, umbilical cord around neck, spinal anesthesia, and perfusion index≥4 were risk factors for poor neonatal prognosis. BMI cannot be used to predict the occurrence of intraoperative hypotension in cesarean section and poor neonatal prognosis, while perfusion index was a potentially valuable indicator of intraoperative hypotension in cesarean section; however, the specificity of perfusion index in poor prognosis of neonates was not high.

The occurrence of nausea and vomiting during cesarean section are important factors that endangers the safety of mother and baby, and the occurrence of hypotension after intraspinal anesthesia is an important factor leading to nausea and vomiting [6, 15, 16]. Mrinalini et al. [17] found that hypotension was an important cause of nausea and vomiting in patients before the delivery of the fetus, and hypotension was the only factor for nausea and vomiting after the delivery of the fetus. Therefore, the prevention and treatment of maternal hypotension during cesarean section has always been the focus of obstetric anesthesia research.

From the results of regression analysis, BMI, infant weight, anesthesia type, puncture site, anesthetic drug dose, and perfusion index were associated with intraoperative hypotension in cesarean section women and poor prognosis of neonates. Cesarean section women with BMI ≥30 kg/m^2^, infant weight ≥3500 g, spinal anesthesia, puncture site L_2-3_, bupivacaine dose>10 mg, ropivacaine dose>50 mg, and perfusion index ≥4 were prone to hypotension symptoms. The reason why overweight women are more prone to hypotension may be that with the increase of maternal BMI, the cerebrospinal fluid solution gradually decreases. In obese patients, epidural vasculature is more engorged and a large amount of fat deposits lead to epidural stenosis [18]. The combined effect of these two factors makes the use of the same dose of local anesthetics during anesthesia also prone to excessive block planes, which ultimately leads to an increased incidence of hypotension. The excessive weight of the fetus may cause the puerperae to compress the inferior vena cava in the supine state, causing in decreased return of blood to the heart, resulting in the occurrence of hypotension [6, 19].

RETRACTED

It has become a consensus that spinal anesthesia is prone to cause maternal hypotension [7, 15, 16]. Clinically, pre-intravenous fluid expansion is often used to prevent hypotension. At the same time, the left 30° supine position is used to move the uterus to the left and vasoconstrictor drugs are given to prevent hypotension. At present, there are studies all over the world reporting the occurrence of hypotension during cesarean section. For example, a study in Ethiopia found that the incidence of maternal hypotension after spinal anesthesia was as high as 64%, and infant weight, spinal induction anesthesia, sensory height block, baseline systolic blood pressure, anesthesiologist experience, and time interval between anesthesia induction and skin incision were risk factors for hypotension after spinal anesthesia [7].

There are few reports on the relationship between the puncture site and hypotension. In our study, in order to make the sensory block level of the patient reach T_6_, the dose of bupivacaine at different puncture sites was different, which may be related to the different incidence of hypotension. Usually, the dose required for spinal anesthesia is relatively small. For general cesarean section, bupivacaine 10 mg or even 7.5 mg can produce a perfect anesthesia effect, and the incidence of hypotension increases significantly when the bupivacaine dose>15 mg. The doses of bupivacaine in our study were mainly distributed between 7 mg and 12 mg, and the incidence of hypotension was 44%.

Perfusion index is currently a new indicator used to predict hypotension in spinal anesthesia for cesarean section. According to a study conducted in India, perfusion index >3.5 is associated with increased risk of hypotension after spinal anesthesia for cesarean section [20]. Similarly, a study in Gansu, China, found that the preanaesthesia pulse variability index (PVI) had a certain predictive value for hypotensive symptoms after epidural anesthesia in cesarean section women [21].

In addition, we also found that risk factors associated with hypotension were associated with poor neonatal prognosis. There are few studies on the effects of the occurrence of hypotension during cesarean section on the fetus. An animal model study showed that fetal bradycardia and acidemia were caused when uteroplacental blood flow was continuously reduced by more than 60% [22]. Hypotension caused by spinal anesthesia is more likely to lead to neonatal acidosis [23]. Short-term hypotension does not affect fetal neurobehavior, while prolonged hypotension can lead to abnormal neonatal neurobehavior [24]. Therefore, vasopressors are usually selected to reduce the adverse effects of hypotension on mothers and neonates.

RETRACTED

The prevention and treatment of hypotension induced by anesthesia during cesarean section has been a focus of clinical research because of the potentially adverse consequences of hypotension on the mother and fetus. The current clinical strategies for the prevention and treatment of hypotension mainly include reducing the dosage of local anesthetics [25], physical assistance method [26], intravenous fluids [26, 27], and using vasoactive drugs [26, 28]. At the same time of prevention and treatment, the combination of risk factor prediction can also reduce the occurrence of hypotension during cesarean section. According to our findings, BMI ≥30 kg/m^2^, umbilical cord around the neck, spinal anesthesia, and perfusion index≥4 are risk factors for poor neonatal prognosis. The existence of high-risk factors may lead to abnormal fetal umbilical arterial blood flow, make the fetus in a state of chronic hypoxia, and ultimately lead to poor perinatal prognosis [29–31].

There are also some shortcomings in this study. First, we did not have data on long-term neonatal follow-up outcomes. Second, further research on these risk factors and the mechanism of hypotension is needed to reduce the incidence of hypotension during cesarean section and improve neonatal prognosis.

## 5. Conclusion

Hypotension is a common complication in cesarean section. Our study found that the prediction model established by BMI, infant weight, anesthesia type, puncture site, anesthetic dose, and perfusion index have certain effect on clinical prediction of hypotension in cesarean section. The prediction model established by BMI, umbilical cord around neck, anesthesia type, and perfusion index have certain guiding value in clinical prediction of poor prognosis of neonates.

## Figures and Tables

**Figure 1:** Flow chart of this study.

**Figure 2:** ROC of BMI and perfusion index for the diagnosis of intraoperative hypotension and poor prognosis of neonates in cesarean section women. (a), ROC for BMI diagnosis of intraoperative hypotension in cesarean section women. (b), BMI diagnosis of ROC with poor neonatal prognosis. (c), ROC of perfusion index for diagnosis of intraoperative hypotension in cesarean section. (d), Perfusion index in diagnosis of ROC with poor neonatal prognosis.

**Table 1:** Clinical data.

Indicators	Total (*n* = 1071)	Indicators	Total (*n* = 1071)
Age (years)	29 (27~32)	Infant weight (g)	3437.33 ± 491.11
BMI (kg/m^2^)	27.82 (23.05~32.35)	Umbilical cord around neck	
Gestational age (week)	39 (38~39)	Yes	161 (15.03%)
Gravidity		No	910 (84.97%)
1~3	908 (84.78%)	1-minute Apgar score	
≥4	163 (15.22%)	≤7	84 (7.84%)
Parity		8-10	987 (92.16%)
1st	625 (58.36%)	Incision direction	
≥2nd	446 (41.64%)	Horizontal	677 (63.21%)
Fetal sex		Vertical	394 (36.79%)
Male	560 (52.29%)	Anesthesia type	
Female	511 (47.71%)	Spinal anesthesia	760 (70.96%)
Hypotension		Epidural anesthesia	311 (29.04%)
Yes	472 (44.07%)	Puncture site	
No	599 (55.93%)	L_2-3_	627 (58.54%)
Fetal position		L_3-4_	444 (41.46%)
Left	713 (66.57%)	Bupivacaine dose (mg)	
Right	358 (33.43%)	≤10	516 (67.89%)
Uterine height (cm)	35 (32, 38)	>10	244 (32.11%)
Abdominal circumference (cm)	105 (98, 112)	Ropivacaine dose (mg)	
Biparietal diameter (mm)	92 (88, 96)	≤50	181 (58.20%)
Femoral length (mm)	72 (68, 76)	>50	130 (41.80%)
Fetal abdominal circumference(mm)	352 (325, 374)	Preoperative HR (times/min)	111 (100, 121)
Anemia		Preoperative MAP (mmHg)	92 (84, 100)
Yes	106 (9.90%)	Intraoperative blood loss (ml)	399 (345, 450)
No	965 (90.10%)	Time from skin incision to delivery (min)	10 (7, 13)
Hypoalbuminemia		Perfusion index	6.47 (3.82, 8.73)
Yes	93 (8.68%)	S/D	2.68 (2.35, 3.20)
No	978 (91.32%)	Amniotic fluid index(mm)	121 (93, 151)

RETRACTED

**Table 2:** Univariate logistic regression analysis of risk factors for intraoperative hypotension in cesarean section women.

Indicators	Control group (*n* = 599)	Hypotension group (*n* = 472)	*χ* ^2^	*p*
Age (years)			0.142	0.706
<35	520 (86.81%)	406 (86.02%)		
≥35	79 (13.19%)	66 (13.98%)		
BMI (kg/m^2^)			21.437	<0.001
<30	423 (70.62%)	269 (56.99%)		
≥30	176 (29.38%)	203 (43.01%)		
Gestational age (week)			0.128	0.720
<37	24 (4.01%)	21 (4.45%)		
≥37	575 (95.99%)	451 (95.55%)		
Gravidity			0.221	0.638
<2	244 (40.73%)	199 (42.16%)		
≥2	355 (59.27%)	273 (57.84%)		
Parity			0.005	0.945
1st	349 (58.26%)	276 (58.47%)		
≥2nd	250 (41.74%)	196 (41.53%)		
Fetal sex			0.483	0.487
Male	307 (51.25%)	252 (53.39%)		
Female	292 (48.75%)	220 (46.61%)		
Fetal position			0.177	0.674
Left	402 (67.11%)	311 (65.89%)		
Right	197 (32.89%)	161 (34.11%)		
Uterine height (cm)			1.983	0.159
<35	266 (4.41%)	230 (48.73%)		
≥35	333 (55.59%)	242 (51.27%)		
Abdominal circumference (cm)			0.446	0.505
<100	184 (30.72%)	154 (32.63%)		
≥100	415 (69.28%)	318 (67.37%)		
Biparietal diameter (mm)			0.004	0.952
<90	202 (33.72%)	160 (33.90%)		
≥90	397 (66.28%)	312 (66.10%)		
Femoral length (mm)			0.001	0.998
<70	203 (33.89%)	160 (33.90%)		
≥70	396 (66.11%)	312 (66.10%)		
Fetal abdominal circumference(mm)			0.030	0.863
<350	290 (48.41%)	226 (47.88%)		
≥350	309 (51.59%)	246 (52.12%)		
Amniotic fluid index (mm)			0.025	0.874
<100	188 (31.39%)	146 (30.93%)		
≥100	411 (68.61%)	326 (69.07%)		
S/D			0.341	0.560
<2.5	221 (36.89%)	166 (35.17%)		
≥2.5	378 (63.11%)	306 (64.83%)		
Anemia			0.022	0.083
Yes	60 (10.02%)	46 (9.75%)		
No	539 (89.98%)	426 (90.25%)		
Hypoalbuminemia			0.434	0.510
Yes	49 (8.18%)	44 (9.32%)		
No	550 (91.82%)	428 (90.68%)		
Infant weight (g)			19.582	<0.001
<3500	385 (64.27%)	240 (50.85%)		
≥3500	214 (35.73%)	232 (49.15%)		
Umbilical cord around neck			0.001	0.994
Yes	90 (15.03%)	71 (15.04%)		
No	509 (84.97%)	401 (84.96%)		
Incision direction			0.512	0.474
Horizontal	372 (62.10%)	283 (59.96%)		
Vertical	227 (37.90%)	189 (40.04%)		
Anesthesia type			21.327	<0.001
Spinal anesthesia	391 (65.28%)	369 (78.18%)		
Epidural anesthesia	208 (34.72%)	103 (21.82%)		
Puncture site			31.152	<0.001
L_2-3_	306 (51.09%)	321 (68.01%)		
L_3-4_	293 (48.91%)	151 (31.99%)		
Bupivacaine dose (mg)	391	369	26.471	<0.001
≤10	300 (76.73%)	219 (59.35%)		
>10	91 (23.27%)	150 (40.65%)		
Ropivacaine dose (mg)	208	103	21.704	<0.001
≤50	127 (61.06%)	34 (33.01%)		
>50	81 (38.94%)	69 (66.99%)		
Preoperative HR (times/min)			0.004	0.951
≤120	447 (74.62%)	353 (74.79%)		
>120	152 (25.38%)	119 (25.21%)		
Preoperative MAP (mmHg)			0.003	0.960
≤90	277 (46.24%)	219 (46.40%)		
>90	322 (53.76%)	253 (53.60%)		
Intraoperative blood loss (ml)			1.232	0.267
≤400	293 (48.91%)	247 (52.33%)		
>400	306 (51.09%)	225 (47.67%)		
Time from skin incision to delivery (min)			2.427	0.119
≤12	413 (68.95%)	346 (73.31%)		
>12	186 (31.05%)	126 (26.69%)		
Perfusion index			256.114	<0.001
<4.0	274 (45.74%)	11 (2.33%)		
≥4.0	325 (54.26%)	461 (97.67%)		

RETRACTED

**Table 3:** Multivariate logistic regression analysis of risk factors for hypotension during cesarean section.

Index	*B*	Std. Error	Wald	df	Sig.	Exp(B)	95% CI	
							Lower bound	Upper bound
BMI ≥30 kg/m^2^	0.680	0.156	19.056	1	<0.001	1.974	1.454	2.678
Infant weight ≥3500 g	0.667	0.151	19.535	1	<0.001	1.949	1.450	2.621
Spinal anesthesia	-0.686	0.16	18.441	1	<0.001	0.504	0.368	0.689
Puncture site L_2-3_	-0.626	0.147	18.116	1	<0.001	0.535	0.401	0.713
Bupivacaine dose >10 mg	0.814	0.16	25.959	1	<0.001	2.258	1.651	3.089
Ropivacaine dose >50 mg	1.157	0.253	20.893	1	<0.001	3.182	1.937	5.227
Perfusion index ≥4.0	3.555	0.318	125.278	1	<0.001	35.005	18.782	65.241

**Table 4:** Univariate logistic regression analysis of risk factors for poor prognosis of neonates.

Indicators	Normal group (*n* = 987)	Poor prognosis group (*n* = 84)	*χ* ^2^	*p*
Age (years)			0.043	0.835
<35	854 (86.52%)	72 (85.71%)		
≥35	133 (13.48%)	12 (14.29%)		
BMI (kg/m^2^)			5.964	0.015
<30	648 (65.65%)	44 (52.38%)		
≥30	339 (34.35%)	40 (47.62%)		
Gestational age (weeks)			3.866	0.049
<37	38 (3.85%)	7 (8.33%)		
≥37	949 (96.15%)	77 (91.67%)		
Gravidity			3.195	0.074
<2	416 (42.15%)	27 (32.14%)		
≥2	571 (57.85%)	57 (67.86%)		
Parity			4.324	0.038
1st	585 (59.27%)	40 (47.62%)		
≥2nd	402 (40.73%)	44 (52.38%)		
Fetal sex			1.335	0.248
Male	511 (51.77%)	49 (58.33%)		
Female	476 (48.23%)	35 (41.67%)		
Fetal position			2.848	0.092
Left	651 (65.96%)	63 (75.00%)		
Right	336 (34.04%)	21 (25.00%)		
Uterine height (cm)			0.063	0.802
<35	456 (46.20%)	40 (47.62%)		
≥35	531 (53.80%)	44 (52.38%)		
Abdominal circumference (cm)			0.377	0.539
<100	314 (31.81%)	24 (28.57%)		
≥100	673 (68.19%)	60 (71.43%)		
Biparietal diameter (mm)			1.679	0.195
<90	339 (34.35%)	23 (27.38%)		
≥90	648 (65.65%)	61 (72.62%)		
Femoral length (mm)			0.016	0.899
<70	334 (33.84%)	29 (34.52%)		
≥70	653 (66.16%)	55 (65.48%)		
Fetal abdominal circumference(mm)			0.121	0.728
<350	474 (48.02%)	42 (50.00%)		
≥350	513 (51.98%)	42 (50.00%)		
Amniotic fluid index (mm)			0.290	0.590
<100	310 (31.41%)	24 (28.57%)		
≥100	677 (68.59%)	60 (71.43%)		
S/D			0.152	0.697
<2.5	355 (35.97%)	32 (38.10%)		
≥2.5	632 (64.03%)	52 (61.90%)		
Anemia			/	/
Yes	882 (89.36%)	83 (98.81%)		
No	105 (10.64%)	1 (1.19%)∗		
Hypoalbuminemia			/	/
Yes	897 (90.88%)	81 (96.43%)		
No	90 (9.12%)	3 (3.57%)∗		
Infant weight (g)			0.055	0.814
<3500	577 (58.46%)	48 (57.14%)		
≥3500	410 (41.54%)	36 (42.86%)		
Umbilical cord around neck			4.107	0.043
Yes	845 (85.61%)	65 (77.38%)		
No	142 (14.39%)	19 (22.62%)		
Incision direction			2.389	0.122
Horizontal	597 (60.49%)	58 (69.05%)		
Vertical	390 (39.51%)	26 (30.95%)		
Anesthesia type			5.787	0.016
Spinal anesthesia	710 (71.94%)	50 (59.52%)		
Epidural anesthesia	277 (28.06%)	34 (40.48%)		
Puncture site			4.144	0.042
L_2-3_	569 (57.65%)	58 (69.05%)		
L_3-4_	418 (42.35%)	26 (30.95%)		
Bupivacaine dose (mg)	710	50	0.340	0.560
≤10	483 (68.03%)	36 (72.00%)		
>10	227 (31.97%)	14 (28.00%)		
Ropivacaine dose (mg)	277	34	0.048	0.827
≤50	144 (51.99%)	17 (50.00%)		
>50	133 (48.01%)	17 (50.00%)		
Preoperative HR (times/min)			0.515	0.473
≤120	740 (74.97%)	60 (71.43%)		
>120	247 (25.03%)	24 (28.57%)		
Preoperative MAP (mmHg)			0.042	0.837
≤90	458 (46.40%)	38 (45.24%)		
>90	529 (53.60%)	46 (54.76%)		
Intraoperative blood loss (ml)			3.022	0.082
≤400	490 (49.65%)	50 (59.52%)		
>400	497 (50.35%)	34 (40.48%)		
Intraoperative hypotension			5.220	0.022
No	562 (56.94%)	37 (44.05%)		
Yes	425 (43.06%)	47 (55.95%)		
Time from skin incision to delivery (min)			7.121	0.008
≤12	702 (71.12%)	43 (51.19%)		
>12	285 (28.88%)	33 (39.29%)		
Perfusion index			8.624	0.003
<4.0	275 (27.86%)	11 (13.10%)		
≥4.0	712 (72.14%)	73 (86.90%)		

∗The number of cases was less than 5, so the data was not included in the final statistics.

RETRACTED

**Table 5:** Multivariate logistic regression analysis of risk factors for poor neonatal prognosis.

	*B*	S.E.	Wald	df	Sig.	Exp(B)	95% CI	
							Lower	Upper
BMI ≥30 kg/m^2^	0.505	0.235	4.613	1	0.032	1.657	1.045	2.627
Gestational age ≥ 37weeks	-0.777	0.446	3.033	1	0.082	0.46	0.192	1.102
Parity≥1	0.455	0.233	3.796	1	0.051	1.575	0.997	2.489
Umbilical cord around neck	0.564	0.285	3.925	1	0.048	1.758	1.006	3.071
Spinal anesthesia	0.616	0.242	6.485	1	0.011	1.851	1.152	2.973
Puncture site L_2-3_	-0.427	0.251	2.897	1	0.089	0.652	0.399	1.067
Intraoperative hypotension	0.198	0.262	0.572	1	0.449	1.219	0.730	2.036
Time from skin incision to delivery>12 min	0.153	0.253	0.365	1	0.546	1.165	0.710	1.912
Perfusion index≥4	0.804	0.366	4.831	1	0.028	2.234	1.091	4.573

## Data Availability

The data used to support the findings of this study are available from the corresponding author upon request.
